# Unsupervised Hyperspectral Microscopic Image Segmentation Using Deep Embedded Clustering Algorithm

This article has been retracted.

**DOI:** 10.1155/2022/1200860

**Published:** 2022-06-06

**Authors:** P. Ajay, B. Nagaraj, R. Arun Kumar, Ruihang Huang, P. Ananthi

**Affiliations:** ^1^Faculty of Information and Communication Engineering, Anna University, Chennai, India; ^2^Department of ECE, Rathinam Technical Campus, India; ^3^Rathinam Technical Campus, Department of Electronics and Communication Engineering, India; ^4^Donghua University, Shanghai, China; ^5^Department of Artificial Intelligence and Data Science, Rathinam Technical Campus, India

## Abstract

Hyperspectral microscopy in biology and minerals, unsupervised deep learning neural network denoising SRS photos: hyperspectral resolution enhancement and denoising one hyperspectral picture is enough to teach unsupervised method. An intuitive chemical species map for a lithium ore sample is produced using *k*-means clustering. Many researchers are now interested in biosignals. Uncertainty limits the algorithms' capacity to evaluate these signals for further information. Even while AI systems can answer puzzles, they remain limited. Deep learning is used when machine learning is inefficient. Supervised learning needs a lot of data. Deep learning is vital in modern AI. Supervised learning requires a large labeled dataset. The selection of parameters prevents over- or underfitting. Unsupervised learning is used to overcome the challenges outlined above (performed by the clustering algorithm). To accomplish this, two processing processes were used: (1) utilizing nonlinear deep learning networks to turn data into a latent feature space (*Z*). The Kullback–Leibler divergence is used to test the objective function convergence. This article explores a novel research on hyperspectral microscopic picture using deep learning and effective unsupervised learning.

## 1. Introduction

Data-driven systems gain knowledge. Recommendations regarding, we need more of them. Data mining, big data, and machine learning are all used. Deep learning without supervision of data classification is a dataset or feature is classified by an application [1]. Data classification is used to make decisions in this circumstance. SVM, linear regression, and feature vectors are examples of data categorization algorithms. This decade, machine learning algorithms have played a critical role in data science. Nonlinear thinking is adapted to real-world problems using machine learning. In ANN (artificial neural network) applications, unsupervised learning is applied. ANN algorithms can learn and comprehend circumstances scientifically thanks to their iterative learning process. Data mining, on the other hand, is a branch of machine learning study that employs unsupervised learning. Predictive models such as SVM, decision trees, and linear discriminant analysis can be used to directly classify data. Even if machine learning for data classification produces improved outcomes, modern application requirements and innovations demand more precision. This new era of study began with the development of deep learning algorithms. Deep learning involves several ANN layers at different levels. So the data is thoroughly analyzed, revealing a huge feature that is transferred to the next layer. The procedure transforms the learnt features from the preceding layer into a high-level data abstraction. Hence, deep learning can be applied to multiclass classification [1, 2].

Many datasets and applications benefit from deep learning, yet its limits open up new research avenues.

1. Deep learning algorithms are supervised learning algorithms. Supervised learning involves labeling or annotating datasets. However, to train and classify for real-time applications, the labeled dataset is expensive and requires a lot of manual labor to manually label
2. Deep learning techniques require a lot of compute to process the huge amount of data. Also, through training on a huge dataset, the deep learning algorithm learns the pattern of comprehension. That is why when talking about deep learning algorithms, CPUs and GPUs come up
3. However, clustering algorithms group data points or features with comparable properties. Unsupervised clustering techniques do this. Unlike supervised deep learning algorithms, it can process grouping and classification without a dataset. Many data applications employ soft or hard clustering methods. Due to the restrictions of the clustering technique, it is difficult to apply it to classification tasks

This study is aimed at improving the behavior and nature of deep learning by using a clustering technique so that deep learning systems can use unsupervised learning to efficiently classify data.

It is widely used to resolve ambiguity. Historical data solves these problems. Algorithms are for supervised machine and deep learning. But unsupervised learning has promise. Experimentation is encouraged. Discriminatory biases are inherent in supervised learning methods, where the set of rules is specified by a set of DOs and DONTs. In the absence of labeling, supervised learning requires a lot of manual work and time.

So the research's major objective is to enhance unsupervised deep learning. Methods for unsupervised learning (b) selecting acceptable and efficient deep learning methodologies and issues to verify and confirm the research findings (d) investigating the best deep learning strategy for data classification. This section's subjects elaborate on the research's goal [3–5].

## 2. Classification Difficulties

A data classification scheme is an integral part of a data security system. Data categorization helps with risk management and data protection. It also offers a natural data hierarchy. Depending on the application, context, content, and behavior, data are employed. Data categorization is used in many ways. In this approach, all segmentation is done manually on tiny datasets. (*b*) Equal intervals: this approach groups data (as desired by the user). (*c*) Quantities: quantity segmentation: a natural break happens when a collection of data changes. It specifies the geometric interval segmentation in each data type. Data are segmented using standard deviation intervals to characterize their attributes and quantify their departure from the normal. (*g*) Custom range: this strategy uses the user's input and may be changed to meet new needs [4, 6].

### 2.1. Implementing Data Classification

1. Manual data classification by their personnel (or in-charges) while storage would be significantly easier: this is not a simple operation if the data is created in large quantities. Today's entities recognize the value of classification and require their process managers to perform it prior to storing. However, their historical data requires modern algorithms and process segmentation/classification
2. The researcher can use several traditional classification approaches, but most are linear and do not work well with data that lacks a pattern. Accuracy varies with dataset size
3. The stated complexity allows for nonlinear techniques like machine learning. But again, machine learning requires labelled data, etc. But the precision is poor
4. The ability of machine learning to operate on unknown data allows for deep learning research. Supervised learning requires a lot of data to train to be effective. Deep learning is important in today's AI. That being said, this platform requires a lot of processing power (GPU) (b) a large labelled dataset preventing over- or underfitting parameters [7, 8]

### 2.2. Implementing Data Classification Strategies

Using a suitable clustering technique, the research is aimed at improving deep learning in an unsupervised mode. The following is the deep learning unsupervised learning approach.

Deep learning is used instead of standard artificial neural networks because it can abstract deep features. The transformation is achieved using a nonlinear deep learning network. *Z* is smaller than *X* due to the transformation. The strategy then processes *Z* to produce *k* clusters by initializing and converging the random centroid. The deep network's clustering and reconstruction losses are determined during this step. It can be trained to minimize loss using the consolidated loss function (LR and LC). Unsupervised learning can be done with the final trained network. For this reason, unsupervised categorization is widely used. The implementation and study are described below [9].

### 2.3. Algorithms for Data

These goals are achieved by unsupervised learning. It looks into clustering methods like *k*-means and FCM. The goal function assigns the data convergent iterative clustering. Clustering loss is crucial in DL networks [10].

DL algorithms are essential in research. To comprehend deep learning algorithms, one must first comprehend ANNs. GDO and thresholding calculations are required. This research begins with autoencoders.

### 2.4. Operational Simulation Tools

TAn open-source Google Brain algorithm is used. That is not all. Applied deep learning requires it. This study uses numpy, pandas, and Scikit-learn to build a model. This research uses MATLAB (mathematical model) [11].

### 2.5. Datasets

It aids in deep learning. Module learning, testing, and validation datasets abound. A WordNet-organized image and vision research dataset is ImageNet. A massive dataset for deep learning, MNIST has 14 million data points. Handwritten NIST digits (7291 training and 2007 testing samples) in 16 × 16 size, quite a dataset. Algorithms for text categorization: this dataset has 80 million CIFAR-10 images in it. Ten classes of 6000 photos each. 50000 records per training and testing set language statistics (STL-10) 96 × 96 photos. They are useless without labels. These datasets are frequently used to validate proposed modules [12].

High-performance imaging applications like superresolution microscopy and cancer detection have made machine learning a potent general tool for scientific data processing: lung cancer diagnostic, human medium expression, and sample classification [13]. Deep learning was used to denoise SRS microscopy and spectra. DeepChem is a sophisticated customized SRS microscopy technology. While DeepChem can segment pictures without spectrally resolved data, it cannot properly identify species without such data. Previously, supervised deep learning was used for CRM image identification. Labeled training data is necessary for DeepChem's spectral resolution and picture and spectrum denoising, while delicate or uncommon biological samples may be collected.

On unsupervised deep learning for CRM image interpretation, unsupervised method finds and segments data. Supervised method: unsupervised model outperforms supervised nonlinear optic signature (HSI). That means it can describe any laser-based optical signal channel, a SRS vibrational spectrum. Other optical microscopy techniques could benefit [14–16].

We SRS-ed each pixel (a). We used two. It took 32 seconds to slice 256 pixels. First, hexadecane and water: C-H stretch resonance 2852 cm^1^ 802 nm pump, 1040 nm Stokes, interval between two beams 92 frames. High- and low-SNR ground truth photos were taken with identical laser input strengths (GT). Due to the high laser power input, hyperspectral, a pixel's local mean and standard deviation (5-pixel radius neighborhood). Using a reference time series, each pixel's PSNR was calculated [16].

Deep learning denoising and segmentation use unsupervised (spodumene, feldspar, and quartz). Its popularity has grown due to the rise of electric cars, AT4O8, where B = boron and T = silicon or aluminum (Al). Like quartz (SiO_2_), a lot of SRS and NOR peaks! The pump beam was 70 mW at 929–998 nm. 909 frames were scanned [16, 17].

### 2.6. NN Models

They both used a neural network. Linked convolutional layer kernel arrays are in conv. Each convolutional layer had this layer (yellow). Encoding required latent space; 4 DE convolutional layer sample size increases with deconvolution. It was used in encoding and decoding (ReLU and leaky-ReLU). The number of fully connected nodes determines a parameter's size [18]. It modifies hyperparameters (hexadecane vs. lithium ore). Identical dataset structure (number and type of layers), a similar validation set optimized the loss. The SI provides model hyperparameters, datasets, and code, that is, supervised or not. It had a good SNR (ground truth). A classic neural network denoiser, our unsupervised method had no supervision. Encoding can only extract properties that are common to many pixels. Our loss was always msd. All pixels were treated as samples during training. Unlike model or hyper parameter data, using one eye improved transferability (supervised method): supervised hyperspectral resolution enhancement (unsupervised hyperspectral resolution enhancement and denoising). Prior algorithms custom PyTorch built on NVidia K80 GPU. It used a ten-layer convolutional auto encoder. It is similar [19].

### 2.7. Autosegmentation

It can classify and denoise spectral components (and, subsequently, image segmentation). Encoding reduces input data dimensionality. A method called *k*-means clustering may find comparable pixels inside an image. This technique is unsupervised, unlike earlier ones. The elbow technique is used in the *k*-means algorithm. The elbow method establishes. The number of components per cluster reduces as *k* grows. The elbow is the inflection point where *k* increases the most. Unsupervised segmentation method: it first projects hyperspectral image data into latent space (blue) (green). This space uses hyperdimensional clustering (*k*-means) to classify each image pixel. The trained autoencoder can automatically identify picture pixels based on hyperspectral properties. Using hyperspectral SRS, each sample constituent is allocated a unique vibrational spectroscopy-based chemical identification [20].

### 2.8. Algorithms for Deep Cluster

Many industries now struggle with data (which has been generated every second in a massive quantity). Deep learning algorithms are essential for research and modernization. Many issues can be solved with supervised learning. However, unsupervised learning may open new doors. But data mining systems' clustering techniques can structure unknown data. Data are clustered using knowledge discovery. Measuring distances is a common clustering: a deep learning and clustering [21] mix.

DEC surplus to unsupervised learning: supervised learning is extended in these ways; algorithms aided DEC core design using autoencoders, and DEC creates a feature space. The clustering technique affects the autoencoder training phase through loss limitations. DEC is a two-stage technique. Pretraining factors like cluster centers and convergence criteria are used to fine-tune the clustering process [22]. This level includes learning and grouping. DEC recommends the autoencoder for data reconstruction since it is simple and reliable (Figure 1). This section introduces DEC and its variants. As stated above, this part is about studying and analyzing algorithms.

Deep learning networks focus on low-dimensional input and learn its features. The autoencoder technique is popular in deep learning networks.

## 3. Loss Function-Deep Clustering

This is because the deep clustering method involves both nonlinear learning and clustering methodology.

### 3.1. Network Loss

Deep learning strategies solely analyze reconstruction loss when using an autoencoder network. Consider the vibrational loss and the adversarial loss when using VAE and GAN. No matter the deep learning network's learning mode, this is required for training (supervised or the unsupervised) [23].

### 3.2. Clustering Loss

A clustering loss that measures algorithm, this study uses them. Adding data points results in a loss. It is estimated using the student *t*-distribution. *k*-means and agglomerative clustering are examples of this loss. It is a clustering loss. And it keeps discriminant information. Group sparsity loss and location loss are discussed [24].

### 3.3. Measuring Results

Metrics for evaluating existing systems and research contributions include measurements that were made using the tagged data from the standard datasets.

#### 3.3.1. Unsupervised Clustering Accuracy (ACC)

The ground truth (*g*) and the clustering assignment output (mp) (c): the unsupervised output has little chance of matching the ground truth labels.

(1) $$\begin{array}{c} \text{ACC}=\text{ma}{\text{x}}_{\text{mp}}\frac{\sum_{j=1}^{n}1\left(g_{j}=\text{mp}\left(c_{i}\right)\right)}{n}, \end{array}$$

where *i* and *j* are loop variables for identifying data points.

#### 3.3.2. Normalized Mutual Information (NMI)

Cluster assignments (*c*) and ground truth labels (*l*) have the same average entropy (*H*) (*g*). This study identifies the output's mutual information compared to the ground truth [25].

(2) $$\begin{array}{c} \text{NMI}\left(g,c\right)=\frac{I\left(g,c\right)}{1/2\left[H\left(g\right)+H\left(c\right)\right]}. \end{array}$$

#### 3.3.3. Adjusted Rand Index (ARI)

ARI calculates the similarity of two data clusters.

The algorithm's success rate is determined by this metric and its assessment. An example of the permutation model is presented below [26].

(3) $$\begin{array}{c} \text{ARI}=\frac{\sum_{ij}^{\text{k}}\left(\begin{array}{c} n_{ij}\\ 2 \end{array}\right)-\left[\sum_{i}^{\text{k}}\left(\begin{array}{c} a_{i}\\ 2 \end{array}\right)\sum_{j}^{\text{k}}\left(\begin{array}{c} b_{j}\\ 2 \end{array}\right)\right]/\left(\begin{array}{c} n\\ 2 \end{array}\right)}{1/2\left[\sum_{i}^{\text{k}}\left(\begin{array}{c} a_{i}\\ 2 \end{array}\right)\sum_{j}^{\text{k}}\left(\begin{array}{c} b_{j}\\ 2 \end{array}\right)\right]-\left[\sum_{i}^{\text{k}}\left(\begin{array}{c} a_{i}\\ 2 \end{array}\right)\sum_{j}^{\text{k}}\left(\begin{array}{c} b_{j}\\ 2 \end{array}\right)\right]/\left(\begin{array}{c} n\\ 2 \end{array}\right)}. \end{array}$$

## 4. Results and Discussion

It was intended to demonstrate our autoencoder networks' image demising and reconstruction abilities. The trained autoencoder networks produced a hyperspectral image from a low SNR image.  Figure 2 shows one shift of 2852 cm^1^ near a peak in hexadecane. The dataset's maximum pixel reading is used to normalize the noisy input image, reducing the perceived dynamic range while resolving the noise. The images clearly reveal two phases, with the hexadecane phase having a stronger signal. SNR may be used to evaluate different neural networks' denoising abilities (Figure 3). The SNR for the GT image in Figure 2 is 31 dB in hexadecane and 10 dB in water. In hexadecane, the SNR is 15 dB, whereas in water, it is 8 dB. We used the model to denoise two new hyperspectral imaging datasets (FOV 1 and FOV 2) for testing. We show examples from 2852 cm^1^ of the denoised hyperspectral dataset. Photos with low SNR are in Figure 4 (20 mW input power).

The GT image was used to compare unsupervised method and supervised method results, not for training. The SNR is 15 dB for unsupervised method, supervised method, and GT and 4 dB for water. Water has an SNR of 86.6 dB, while hexadecane is 14. They both use spectral data to improve picture quality.  Figure 2 shows a 15 m droplet in the FOV 2 ROI. It also shows more defined droplet boundaries. The PSNR of noisy GT data is 14, unsupervised method is 22, and supervised method is 25 dB [27].

Peak resolution is critical for SRS component categorization. Supervised method and unsupervised method denoise images across the entire spectrum (Figure 2). Supervised method denoises SRS spectra using a trained model on an unknown dataset. Figure 4 shows a low SNR image of hexadecane water with a spectrum around the C-H stretch. As shown in Figure 4, the supervised method output spectrum (red) is represented by a pixel in Figure 5. SNR GT spectrum (green) is in Figure 4 (60 mW input power). Suppressing GT data from input, supervised method, and unsupervised method spectra reduced spectral noise. Figure 5 shows the input, supervised method, and unsupervised method residuals for a pixel. To compute PSNR, we use the GT as a reference in Figures 4 and 6. The water-hexadecane phase boundary moved between high- and low-SNR recordings (60 mW input power). The input PSNR is 12.1 dB, while the supervised method output is 23.2 dB. Both processing methods improve hyperspectral contrast and reduce noise in unsupervised method [28].

SRS datasets often contain “stitched” spectral scan spectra. These two phenomena are nonlinear optical phenomena. The unsupervised method was tested on a complex lithium ore sample. Weak linear absorption reduces sample power. In this sample, the diversity reduces collected signal. In a spectral focus scan, the SRS vibrational spectrum shows the Pump-Stokes delay. We also offer hyperspectral index maps (blue). Noisy image data unsupervised method model on lithium ore is not shown. Its output (red) is shown in Figure 5(a). This method improves SNR while maintaining spectral resolution, less spectral resolution and peak contrast. Then, a 10-pixel average filter (blue), smoothing reduces peak contrast and spectral resolution (b). A high absorption semiconductor material (pyrite) may be present in these mineral samples [29].

The encoder's latent space can be segmented using clustering. Compare directly with known mineral complex spectra [30]. Non-SRS modulation transfer signals are automatically segmented using *k*-means because they are saturated at the detector. Ingredient-specific unsupervised single-pixel spectra compared to Ref. (black dashed lines). These are the model's spectra. In this case, unsupervised + *k*-means works well. Easily create chemical species maps from images.

The proposed algorithm and FCM versions are tested on 300 samples from various datasets. The results were tested with both Table 1 noisy data and Figure 2 noiseless images to assess the proposed algorithm's property handedness. In the noisy mode of analysis, DEC outperforms other descendants of the FCM (except specific sample).  Table 2 and Figure 2 show the proposed DEC comparison result.

The same comparison procedure with noiseless data in Table 3 and Figure 6 compares the DEC and FCM versions. The proposed DEC outperforms the other algorithms. In both noisy and quiet environments, the proposed DEC performs well (Figure 7). For the noise sensitivity test, the image was processed with various noise variances (such as 0.2, 0.4, 0.6, and 0.8).

## 5. Conclusion

In this work, deep learning was employed to improve contrast and identify chemical species. Index variable for any laser parameter, TL or CPM microscope spectra examples of SRS vibrational spectra SRS contrast enhancement supervised and unsupervised spectra (the latter recorded at high SNR). *k*-means clustering for unsupervised picture segmentation, this chemical species map has several applications. Harmonic generation, fluorescence, and thermal lensing are a few examples. Unsupervised picture denoising and material identification are available globally. Deep learning complements dimension reduction methods effectively. As a preprocessing unit, fraternal *K*-median clustering maintains and enhances the important information available in and via regularization utilizing dropout approach. But even if the dropout probability is larger, the SH-FE techniques are vital in boosting cluster values. The findings and discussions show that the technique devised offers the best outcomes in terms of time complexity and accuracy.

## Figures and Tables

**Figure 1:** Deep clustering networks with stacked autoencoder.

**Figure 2:** Microscopic dataset list.

**Figure 3:** Contingency matrix table.

**Figure 4:** Microscopic segmented dataset list.

**Figure 5:** Comparison of clustering algorithms (for noisy data).

**Figure 6:** Clustering algorithms for noiseless data comparison.

**Figure 7:** Clustering algorithms for noisy variance data comparison.

**Table 1:** Noisy data comparison on clustering algorithms.

Data	FCM	FCM_S	En-FCM	FLICM	M-FLMCM	Proposed DEC
I1	62.71	72.30	67.22	75.25	81.25	83.10
I2	62.90	71.55	67.95	76.63	81.10	83.38
I3	61.85	73.82	67.12	75.53	80.01	82.86
I4	62.95	74.16	66.97	74.51	79.46	83.16
I5	60.98	70.80	67.86	74.58	78.75	82.25

**Table 2:** Noiseless data comparison on clustering algorithm.

Data	FCM	FCM-S	En-FCM	FLICM	M-FLMCM	Proposed DEC
I1	84.53	84.88	84.99	82.74	84.89	89.026
I2	83.81	83.52	84.28	82.13	84.56	82.726
I3	83.21	82.07	81.40	82.34	84.57	90.811
I4	82.24	84.79	84.13	82.91	84.31	83.563
I5	81.90	83.96	84.00	82.19	82.33	84.999

**Table 3:** Noisy variance data comparison on clustering algorithms.

Noise variance	FCM	FCM_S	En-FCM	FLICM	M-FLMCM	Proposed DEC
0.2	81.80	83.16	82.15	83.26	83.62	84.26
0.4	78.08	76.12	78.30	78.97	76.06	79.50
0.6	71.91	73.59	71.70	72.25	71.97	75.00
0.8	68.70	67.53	67.44	66.52	67.39	70.77

## Data Availability

The data used to support the findings of this study are available from the corresponding author upon request.

## References

[1] Ren Y., Hu K., Dai X., Pan L., Hoi S. C., Xu Z. (2019). Semi-supervised deep embedded clustering. *Neurocomputing*.

[2] Xie J., Girshick R., Farhadi A. Unsupervised deep embedding for clustering analysis.

[3] Zhang Y., Kang L., Wong I. H. (2022). High-throughput, label-free and slide-free histological imaging by computational microscopy and unsupervised learning. *Advanced Science*.

[4] McRae T. D., Oleksyn D., Miller J., Gao Y. R. (2019). Robust blind spectral unmixing for fluorescence microscopy using unsupervised learning. *PLoS One*.

[5] Pattanaik P. A., Mittal M., Khan M. Z. (2020). Unsupervised deep learning cad scheme for the detection of malaria in blood smear microscopic images. *IEEE Access*.

[6] Du X., Dua S. (2010). Segmentation of fluorescence microscopy cell images using unsupervised mining. *The Open Medical Informatics Journal*.

[7] Yu H., Guo D., Yan Z. (2018). Unsupervised learning for large-scale fiber detection and tracking in microscopic material images.

[8] Purwar Y., Shah S. L., Clarke G., Almugairi A., Muehlenbachs A. (2011). Automated and unsupervised detection of malarial parasites in microscopic images. *Malaria Journal*.

[9] Sahare S., Ghoderao S., Yin P. (2022). An Assessment of MXenes through Scanning Probe Microscopy. *Small Methods*.

[10] Xing F., Xie Y., Su H., Liu F., Yang L. (2018). Deep learning in microscopy image analysis: a survey. *IEEE Transactions on Neural Networks and Learning Systems*.

[11] Wang X., Li J., Ha H. D. (2021). AutoDetect-mNP: an unsupervised machine learning algorithm for automated analysis of transmission electron microscope images of metal nanoparticles. *Jacs Au*.

[12] Binnig G., Rohrer H. (1983). Scanning tunneling microscopy. *Surface science*.

[13] Revilla-León M., Gohil A., Barmak A. B. Influence of ambient temperature changes on intraoral scanning accuracy. *The Journal of Prosthetic Dentistry*.

[14] Speiser A., Turaga S. C., Macke J. H. (2019). Teaching deep neural networks to localize sources in super-resolution microscopy by combining simulation-based learning and unsupervised learning. https://arxiv.org/abs/1907.00770.

[15] Shu C., Chen X., Xie Q., Han H. (2018). An unsupervised network for fast microscopic image registration. *Medical Imaging 2018: Digital Pathology*.

[16] Chen X., Velliste M., Murphy R. F. (2006). Automated interpretation of subcellular patterns in fluorescence microscope images for location proteomics. *Cytometry Part A: The Journal of the International Society for Analytical Cytology*.

[17] Dave I. R., Upla K. P. Computer aided diagnosis of malaria disease for thin and thick blood smear microscopic images.

[18] Lu A. X., Kraus O. Z., Cooper S., Moses A. M. (2019). Learning unsupervised feature representations for single cell microscopy images with paired cell inpainting. *PLoS Computational Biology*.

[19] Liu D., Zhang D., Song Y. (2021). Pdam: a panoptic-level feature alignment framework for unsupervised domain adaptive instance segmentation in microscopy images. *IEEE Transactions on Medical Imaging*.

[20] Masubuchi S., Machida T. (2019). Classifying optical microscope images of exfoliated graphene flakes by data- driven machine learning. *npj 2D Materials and Applications*.

[21] Liu D., Zhang D., Song Y. Unsupervised instance segmentation in microscopy images via panoptic domain adaptation and task re-weighting.

[22] Xin T., Chen B., Chen X., Han H. UTR: unsupervised learning of thickness-insensitive representations for electron microscope image.

[23] Regina A. A. (2015). Detection of leukemia with blood microscopic images. *Journal of Innovative Research in Computer and Communication Engineering*.

[24] Duggal R., Gupta A., Gupta R., Wadhwa M., Ahuja C. Overlapping cell nuclei segmentation in microscopic images using deep belief networks.

[25] Baltissen D., Wollmann T., Gunkel M. Comparison of segmentation methods for tissue microscopy images of glioblastoma cells.

[26] Agaian S., Madhukar M., Chronopoulos A. T. (2014). Automated screening system for acute myelogenous leukemia detection in blood microscopic images. *IEEE Systems Journal*.

[27] He S., Minn K. T., Solnica-Krezel L., Li H., Anastasio M. (2019). Automatic microscopic cell counting by use of unsupervised adversarial domain adaptation and supervised density regression. *Medical Imaging 2019: Digital Pathology*.

[28] Riccio D., Brancati N., Frucci M., Gragnaniello D. (2019). A new unsupervised approach for segmenting and counting cells in high-throughput microscopy image sets. *IEEE Journal of Biomedical and Health Informatics*.

[29] Ta V. T., Lezoray O., Elmoataz A. Graph based semi and unsupervised classification and segmentation of microscopic images.

[30] Li W., Field K. G., Morgan D. (2018). Automated defect analysis in electron microscopic images. *npj Computational Materials*.

